# Open Partial Nephrectomy in Renal Cancer: A Feasible Gold Standard Technique in All Hospitals

**DOI:** 10.1155/2008/916463

**Published:** 2008-08-26

**Authors:** J. M. Cozar, M. Tallada

**Affiliations:** Department of Urology, Virgen de las Nieves University Hospital, Granada, Spain

## Abstract

*Introduction*. Partial nephrectomy (PN) is playing an increasingly important role in localized renal cell carcinoma (RCC) as a true alternative to radical nephrectomy. With the greater experience and expertise of surgical teams, it has become an alternative to radical nephrectomy in young patients when the tumor diameter is 4 cm or less in almost all hospitals since cancer-specific survival outcomes are similar to those obtained with radical nephrectomy. *Materials and Methods*. The authors comment on their own experience and review the literature, reporting current indications and outcomes including complications. The surgical technique of open partial nephrectomy is outlined. *Conclusions*. Nowadays, open PN is the gold standard technique to treat small renal masses, and all nonablative techniques must pass the test of time to be compared to PN. It is not ethical for patients to undergo radical surgery just because the urologists involved do not have adequate experience with PN. Patients should be involved in the final treatment decision and, when appropriate, referred to specialized centers with experience in open or laparoscopic partial nephrectomies.

## 1. INTRODUCTION

In recent years, the surgical treatment of renal cell carcinoma (RCC) has developed towards conservative surgery of the renal parenchyma and the use of minimally invasive techniques. The emerging conservative technique is open partial nephrectomy (PN), which is no longer an option reserved for patients with a single kidney or bilateral renal tumors; it has become a viable alternative to radical nephrectomy, and is considered the treatment of choice for selected patients with a normal contralateral kidney [1, 2].

The more frequent use of PN in renal cancer treatment derives from a spectacular rise in the incidental diagnosis of renal tumors in patients undergoing abdominal ultrasound or computed tomography (CT) for abdominal diseases. This has markedly increased the detection of smaller, asymptomatic tumors than those observed when Robson proposed radical nephrectomy as the technique of choice more than three decades ago [3]. Incidental tumors have a more favorable prognosis than clinically detected or symptomatic tumors of a similar size and stage [4, 5]. The better health and longer life span of the general population and the availability of radiological imaging techniques for closer screening and follow-up programs are creating a favorable environment for the development of conservative renal surgery. When PN is indicated, the decision to adopt an open or laparoscopic (minimally invasive) approach depends on the benefits and risks to the patient and the experience of the surgical team.

This article is devoted to open PN, providing an update on the indications, disease-free and disease-specific survival outcomes, benefits and risks, limitations and technical aspects of the surgery, intra- and postoperative complications, and post-treatment follow-up protocols. The aim is to describe the main concepts to be considered in the decision-taking algorithm for an open PN in the treatment of RCC [6, 7].

## 2. INDICATIONS FOR PARTIAL NEPHRECTOMY

Indications can be classified as absolute, relative, or elective (Algorithm 1), always basing the selection on the viability of the technique and an optimal cancer control [8].

### 2.1. Absolute indications

Absolute indications relate to patients who would be anatomically or functionally anephric if radical nephrectomy was performed. They include the presence of only one kidney, synchronous bilateral renal cancer, and severe renal failure. It was proposed in the 1950's that these patients undergo conservative tumor excision to preserve maximum renal parenchyma and allow the possibility of renal filtration with no need for dialysis. However, this proposal gained little acceptance among urologists due to the high rate of complications observed after open PN. More recently, there has been a strong resurgence in the use of this technique as an alternative to radical nephrectomy for the above-mentioned types of patients. In the 1990's, various studies reported good survival outcomes and fewer complications with a conservative approach.

### 2.2. Relative indications

These include conditions that might compromise the future functioning of the contralateral kidney (without tumor), for example, moderate renal failure, nephrolithiasis, recurrent pyelonephritis with parenchymal lesions, vesicoureteral reflux, and congenital or acquired obstruction of the urinary tract, among others. A further relative indication would be the presence of disease with a potentially negative medium-term effect on renal function, for example, diabetes or hypertension. Other factors must be taken into account in these patients, including their current age and age at onset of the disease, estimating the duration of its possible effect on renal function.

### 2.3. Elective indications

Partial nephrectomy has been proposed for small peripheral renal tumors over the past few years. Being initially controversial, this indication has been supported by wide studies showing similar outcomes to radical surgery in small (≤4 cm) renal tumors (Algorithm 1). The age and general state of the patient are important in the selection of candidates for PN, which is most beneficial for young and healthy patients. Some authors have proposed to widen the indication for a conservative approach to include larger tumors of up to 7 cm. Thus, Fergany et al. at the Cleveland Clinic reported similar five-year disease-free survival rates between patients with tumors <4 cm and those with tumors of 4–7 cm [4].

The greater longevity of the population and the treatment of ever younger patients for incidentally detected tumors have drawn attention to the long-term risks of renal failure or metachronous tumor recurrence posed by PN treatment. Nevertheless, these risks should not outweigh the benefits of this renal parenchyma-preserving surgery.

## 3. CLINICAL EXPERIENCE: SURVIVAL OUTCOMES

There is now considerable clinical experience in patients with one of the above indications for PN, allowing careful analysis of patient outcomes and evaluation of the prognostic factors that influence results.

Studies of patients with small renal tumors at the Memorial Sloan Kettering Cancer Center of UCLA, Mayo Clinic, and Cleveland Clinic showed no significant differences in five-year survival rates (91–100%) between those treated with open PN and those treated with open radical nephrectomy (Figure 1) [9–14]. Long-term follow-up studies have corroborated these results. Thus, Lau et al. compared between patients treated with open PN (mean tumor size of 3.7 cm) and those treated with radical nephrectomy (mean size of 3.3 cm), and found no significant differences in overall survival, cancer-specific survival, metastasis-free survival, or local recurrence-free survival at 5, 10, or 15 years [11]. These findings validate the oncological efficacy of conservative versus radical renal surgery.

There have been no prospective randomized clinical trials comparing the two techniques. Moreover, global results of the published studies cannot be grouped together because the distribution of indication levels (absolute, relative, or elective) is different in each study population. For this reason, outcomes of open PN are reported below in relation to the type of indication.

### 3.1. Outcomes of partial nephrectomy with absolute indication

In general terms, patient survival rates are lower when the indication for surgery is absolute rather than elective, influenced by the higher age, the more advanced stages, the larger tumor size, and the poorer health status of patients with an absolute indication. Reports from the Cleveland and Mayo Clinics [4, 15] described disease-free survival rates after PN of 81–88% at 5 years and 64–73% at 10 years, being relatively similar to disease-free survival rates described for radical nephrectomy in tumors of the same size and stage. In 2007, Berdjis et al. studied 38 cases of open PN in single kidney carried out between 1993 and 2003 [16]. After a mean follow-up of 41.7 months, they observed local recurrence in four patients (including 3 with distant progression) and metastatic progression in two. Tumor size was significantly larger in patients with metastatic progression versus those without (6.2 cm versus 3.5 cm) and in patients with subsequent renal failure versus those without (5.2 cm versus 3.3 cm).

According to these authors, tumor size is the most significant prognostic factor for disease progression followed by tumor stage (localized versus locally advanced), and larger tumor size is the main prognostic factor for renal failure onset [16].

### 3.2. Results of partial nephrectomy with elective indication

In the 1990's, numerous reports [5, 10, 11, 17–26] were published on a total of 572 patients with normal contralateral kidney treated by open PN, having tumor sizes ranging from 2 to 4.3 cm (Table 1). A survival rate of 90–100% was achieved in these cases, with a local recurrence rate of 0% in most series [10, 11, 18–20–25, 27], 1% in 2 series [5, 22], 3% in 2 series [12, 21], and 6-7% in 2 series [13, 26]. These outcomes opened up the way for open PN to become an effective alternative to radical nephrectomy although higher rates of intra- and postoperative complications were initially observed.

Published data establish 4 cm as the cut-off tumor size for indication of this surgery, describing a shorter disease-free survival period in patients with larger tumors. Studies report 95% five-year disease-free survival rates in patients with a tumor <4 cm, comparable to the outcomes of radical nephrectomy in tumors of a similar size (Table 1).

### 3.3. Results of partial nephrectomy in patients with Von Hippel Lindau (VHL) syndrome

The risk of local recurrence is very high in VHL patients because of the multifocal nature of their malignant tumors; consequently their disease-free survival is much lower in comparison to patients with incidental or sporadic renal carcinoma.

Out of nine VHL patients with bilateral renal carcinoma studied by Novick and Campbell, seven had local recurrence and one died from metastatic disease [2]. It is likely that most of these recurrences represented a manifestation of a microscopic residual CCR that was not excised during the NP [2].

Walther et al. [27] reported on 52 VHL patients with renal cancer treated at the National Cancer Institute, finding that no patient with tumors <3 cm developed metastatic disease. They therefore recommend waiting until this type of tumor reaches 3 cm in order to reduce the need for surgery before onset of the multiple recurrences observed during follow-up of these patients.

The effectiveness of PN as a valid alternative for the treatment of this disease was demonstrated by a multicenter study in USA on the results of treating 65 patients with VHL and localized RCC (54 bilateral, 11 unilateral). PN was performed on 49 of these patients, with five-year and ten-year survival rates of 100% and 81%, respectively. These survival outcomes are similar to those obtained with radical nephrectomy, and they support the role of PN in the treatment of this type of patient.

In patients with advanced VHL and large multiple bilateral tumors that require complete excision of both kidneys at first surgery or after various interventions due to the post-PN growth of residual RCCs, renal transplant is an appropriate option to avoid terminal kidney failure and the need for dialysis, especially in young patients with this genetic syndrome.

## 4. PROGNOSTIC FACTORS FOR TUMOR RECURRENCE AFTER PARTIAL NEPHRECTOMY

In RCC, prognostic factors for distant recurrence or metastatic progression after radical nephrectomy are known to include the Fuhrman grade, size, and stage, as well as histological type of the tumor, the presence of positive lymph nodes, and ECOG performance status [2, 8]. Some of these factors, described below, are of special interest in selecting candidates for PN.

### 4.1. Tumor size >4 cm

Tumor size was found to be the most significant predictor of the outcome in large series of PN patients [4, 11, 13, 25]. Tumor size independently predicts local recurrence and is the most important criterion for the indication of a PN. The Cleveland Clinic series of 485 PNs, including 9% with elective indications, showed significant differences in five-year and ten-year survival rates between patients with tumors smaller and larger than 4 cm, with a significant correlation between recurrence rate and tumor size. For this reason, Barbalias et al. [25] proposed a subclassification of stage T1 (tumors <7 cm and limited to renal parenchyma) into T1a and T1b for tumor sizes of <4 cm and ≥4 cm, respectively.

Lerner et al. [13] observed a 95% five-year survival rate in PN patients with tumors <3 cm versus an 80% rate in those with tumors >6 cm. They also reported a significantly higher disease-free survival rate in patients with tumors >4 cm after radical versus partial nephrectomy. More recently, various studies [9–14, 23] (Figure 2) demonstrated equivalent cancer control rates between patients with tumors <4 cm and those with tumors of 4–7 cm after electively indicated PN.

### 4.2. Localization of tumor

It was classically thought that centrally localized tumors carried a greater risk of metastasis at the time of disease presentation. It was therefore considered that the risk of recurrence and/or progression would be higher after partial versus radical nephrectomy in central tumors. This idea was challenged by the results of a retrospective study by D'Armiento et al. [23] on tumor localization as an independent risk factor. They found no difference in cancer-free survival or recurrence between peripheral tumors (not extending into the interior of the kidney) and central tumors (infiltrating beyond the renal medulla). These authors concluded that PN is more complex in the case of central tumors, but it is not associated with a worse recurrence or progression prognosis.

### 4.3. Multifocality

The incidence of small renal tumors removed during radical nephrectomy for RCC or in necropsies ranges from 4 to 25% [27, 28]. As a consequence, many urologists have argued against PN as a standard treatment for RCC, even when tumors are small, due to the high risk of multifocality. We need to know the factors that increase the risk of multifocality to allow us to select PN when the risk of multifocality is low and radical nephrectomy when the risk is high.

The main factor signaling an increased risk of multifocality is large tumor size, since 91% of multifocal tumors are associated with primary tumors >5 cm [29]. The second factor is tumor stage (pT2 or higher). Thus, stage pT3a shows a 16.4% incidence of multifocality, with a mean distance between primary and secondary tumors of 26.4 mm [30]. Other factors increasing the risk of multifocality cannot be known before surgery but only after examination of the surgical specimen, including histological factors such as vascular infiltration and papillary or mixed histological variants [27]. Knowledge of factors carrying an elevated risk of multifocality alerts to the need for more rigorous patient follow-up and inspection of the whole defatted kidney to rule out satellite tumors during PN.

With regard to the preoperative detection of multifocal lesions by imaging techniques, only 22.9% of additional tumors subsequently observed in specimens after radical nephrectomy had been detected by ultrasound or CT [31]. Intraoperative ultrasound studies show a higher sensitivity, detecting up to 78% of multifocal tumors, which may be very useful when there are multifocality risk factors and a PN has been proposed to the patient.

### 4.4. High Fuhrman nuclear grade and symptomatic clinical presentation

It was reported that recurrence-free survival after PN was not only significantly improved by smaller tumor size (<4) but also by low Fuhrman grade and incidental clinical presentation [4]. This finding was confirmed by Licht [32], who observed a significantly worse prognosis after this surgery in symptomatic (83% five-year survival) versus incidental (94% five-year survival) tumors.

Moll et al. [5] and Ghavamian et al. [15] reported that tumor stage and nuclear grade are significantly associated with RCC mortality. These classic prognostic factors are valid for both radical and partial nephrectomies, but a much more rigorous follow-up is required if partial nephrectomy is selected and the pathology study reports grade III disease.

### 4.5. Surgical margins

Conventional PN includes ≥1 cm margin of healthy parenchyma, whereas this margin is not left in tumor enucleation and there is a higher risk of surgical margin involvement. Recent reports have shown similar rates of cancer control between PN and enucleation, provided that surgical margins in enucleation are examined by intraoperative biopsy of the kidney bed.

In a series of 44 patients treated with PN for tumors with a mean size of 3.2 cm and a mean surgical margin of 2.5 mm, 93% had negative surgical margins and showed no local recurrence after a mean follow-up of 4 years [33]. In the Mayo Clinic series, all partial nephrectomies were carried out with margins ≥3 mm of healthy peritumoral renal tissue, verified by intraoperative biopsy of the kidney bed. Local five-year recurrence-free survival was 97% in a series of 130 patients [34].

It can therefore be proposed that a margin of 1-2 cm is not necessary in PN, for which a few millimeters (3–5 mm) can be adequate as long as the intraoperative biopsy of the kidney bed is negative.

## 5. SURGICAL TECHNIQUE IN PARTIAL NEPHRECTOMY

Surgical technique in PN has advanced over recent years, offering improved cancer control and anatomical-functional outcomes for the saved kidney.

A flank incision approach is used, opening Gerota's fascia and localizing the kidney and the tumor. A thorough visual inspection is essential for adequate planning of the resection, especially if the tumor is near the hilum. It is controversial whether renal ischemia is required for the resection. This decision depends on the nature of the tumor and the skill of the surgeon. At our center, where there is considerable experience acquired over many years and excellent cancer control and renal preservation outcomes have been obtained, the renal pedicle is identified and released, isolating the main renal artery and vein with vessel-loops.

If the tumor is small and the indication is elective, resection of the tumor then commences, allowing a safety margin of several millimeters of healthy renal parenchyma. If there is no major bleeding as the resection proceeds, total resection of the tumor is completed without recourse to any type of renal ischemia. If there is any doubt about the resection margins after removal of the tumor, an intraoperative biopsy of the bed is performed and we proceed according to the results. Then, hemostasis of the tumor bed is started rapidly with single stitches of 4/0 vicryl at the main bleeding points using spray-coagulation on secondary vessels with an electric scalpel, which takes considerable time. To reduce this time, a technique modification was introduced at our centre one year ago, with the application of a fibrinogen hemostatic patch (Tachosil, Nycomed Pharma, Austria) on the resection surface after suturing the main bleeding vessels. This has shortened the time for intervention and hemostasis to 15–20 minutes, and improved the visual appearance (Figure 3). We also leave the surgical bed open after the resection, without using a mattress stitch to draw the renal parenchyma together for better hemostasis. The resection bed must be carefully inspected, and the opening of the urinary passage (calyx or pelvis) must be avoided or, when necessary, repaired.

When tumors are large but PN is relatively or absolutely indicated, we prefer to clamp the renal artery to produce ischemia after administering intravenous mannitol, keeping the renal vein patent to minimize the risk of postoperative acute tubular necrosis. It may also be necessary to clamp the renal artery in cases of central tumors that affect major vessels (e.g., arcuate arteries) or in cases of unexpected bleeding that can only be controlled by ischemia. In these cases, it is very useful to have the renal pedicle prepared in advance, allowing ischemia to be produced within a few seconds and minimizing blood loss.

Intraoperative ultrasonography is not a standard procedure in our setting but can greatly assist in the identification of other renal tumors when multifocality is suspected. Some authors use intraoperative ultrasonography to demarcate intrarenal tumors and to avoid damaging large vessels near the resection line or bed.

Once hemostasis has been achieved, a careful examination is required to detect any inadvertent opening of the urinary tract, thereby avoiding postoperative leaks or fistulas. If an opening is identified, it is closed using a resorbable suture. When an opening is suspected but cannot be seen, an intrapelvic injection of methylene blue is required, leading some authors to previously insert a ureteral stent in patients with central-located tumors. Fibrin sealants, as well as being hemostatic agents, can reinforce repair of the collecting system. Gelfoam soaked with thrombin can be placed over the defect and then infiltrated with Hemaseel fibrin sealant to close small defects of the urinary tract at the level of the calyces.

## 6. COMPLICATIONS OF OPEN PARTIAL NEPHRECTOMY

Open partial nephrectomy is more complex than radical nephrectomy, and many authors place limits on its use citing a higher risk of complications. Several decades ago, reports on open PN described a greater risk of acute renal failure, urinary fistula, and hemorrhage of the surgical bed, among other complications [15, 22, 35, 36].

The lower incidence of complications in the present patient series can be attributed to the greater experience that urologists have gained with this technique and the higher prevalence of incidental small tumors. In 1994, Campbell et al. [35] described complication rates after open PN of 37% for symptomatic tumors and of 22% for incidental tumors Table 2.

More recently, however, open PN and radical nephrectomy have shown a similar complications' rate, overall morbidity rate, hospital stay, blood losses, and frequency of acute renal failure [37, 38]. The risk of acute renal failure after open PN ranges from 0 to 18% according to the series. Campbell et al. [35] reported a 13% incidence of acute renal failure in 259 patients after open PN (for which only 10/259 patients [3.9%] had an elective indication). Risk factors for postoperative acute renal failure were tumor size >7 cm, excision of more than half the renal parenchyma, and ischemia >60 minutes. In patients with PN, the renal parenchymal volume loss correlates best with the renal function loss several months after surgery. Estimates of volume loss may be useful for predicting postoperative renal function when planning PN in patients with a solitary kidney [6, 7, 39].

The risk of urinary fistula after open PN ranges from 1.8 to 21%, and is lower in patients treated for a small incidental tumor with elective indication. Campbell et al. [35] described an increased risk of urinary fistula in tumors >4 cm localized centrally or near the hilum in surgery requiring reconstruction of the excretory tract.

To summarize, complications of open PN appear to have been reduced to levels found with open radical nephrectomy—thanks to the greater experience of surgical teams with this technique. In the medium term, however, at 6–12 months, open PN patients have a significantly lower serum creatinine level compared with laparoscopic radical nephrectomy patients [40]. This information must be explained to patients when they are informed about the short-term and long-term risks of the two approaches.

## 7. FOLLOW-UP GUIDELINES AFTER OPEN PARTIAL NEPHRECTOMY

Several clinical guidelines have been established for the follow-up of patients after open PN, based on detailed analysis of reported tumor recurrence patterns at specialized centers (e.g., Cleveland Clinic).

Rates of local recurrence and metastatic progression vary as a function of the tumor stage at surgery as follows: T1N0M0: 0% local recurrence and 4.4% distant progression; T2N0M0: 2% and 5.3%, respectively; T3aN0M0: 8.2% and 11.5%, respectively; T3bN0M0: 10.6% and 14.9%, respectively. Postoperative time periods associated with a maximum incidence of local recurrence are between 6 and 24 months for T3 and T2 tumors and after 48 months for T1 tumors. Hence, the follow-up time and protocol are selected according to the pathological stage at the time of the open PN.

Novick and Campbell [2] proposed these follow-up guidelines.

1. Patients with T1N0M0 tumors have annual anamnesis, physical examination, and serology, with no need for radiology during the first year. No subsequent systematic diagnostic imaging studies are required due to the low risk of recurrence.
2. Patients with T2N0M0 tumors have annual anamnesis, physical examination, chest X-ray, and abdominal CT scan, with abdominal X-ray every 2 years.
3. Patients with T3N0M0 tumors have anamnesis, physical examination, chest X-ray, and abdominal CT every 6 months for 3 years and then annually.

In the long term, hyperfiltration can cause renal injury in these patients, especially if there has been >50% loss of nephrons, with proteinuria, focal segmental glomerulosclerosis, and progressive renal failure. Because proteinuria is the first change in this disorder, 24-hour urine proteins should be determined annually in all patients with suspicion of hyperfiltration due to loss of renal parenchyma.

## 8. WHEN TO PROPOSE OPEN PARTIAL NEPHRECTOMY

Based on the above reported data, clinical studies (Mayo Clinic, Cleveland Clinic, UCLA, etc.), and our own experience, we can affirm, in common with other authors [1, 2], that open PN is now the gold standard treatment for young and healthy patients with incidentally detected small renal tumors (<4 cm). It also represents an alternative to radical nephrectomy in single-kidney patients or those with bilateral tumors.

The presence of renal failure, diseases that predispose towards renal failure, or genetic syndromes associated with multifocality also shows indications for open PN versus radical nephrectomy since, in small tumors, there are no differences in disease-free survival, morbidity, or complication rates between the techniques.

The current standard surgical technique for partial nephrectomy is open partial nephrectomy. Only certain highly specialized centers have gained sufficient experience with laparoscopic PN to minimize its risks and complications [40]. It remains a challenging technique, requiring a longer period of warm renal ischemia, vein closure, and the difficult suturing of open vessels during tumor resection. In fact, the laparoscopic approach has been associated with a higher rate of complications, even in the best hands. Thus, Sharma et al. reported intra- and postoperative complication rates of 5% and 11%, respectively, using laparoscopic PN, compared with 0% and 2%, respectively, using open PN [39].

Although no studies have been published to date on the long-term oncological effectiveness of laparoscopic PN [1], preliminary data indicate that it does not differ from that obtained with the open approach. In 2007, Gill et al. [41] reported three-year cancer-specific survival rates of 99.3% in 771 patients treated with laparoscopic partial nephrectomy and 99.2% in 1028 patients treated with open partial nephrectomy. The same study confirmed a shorter surgery time (*P* < .0001), hospital stay (*P* < .0001), and a lower blood loss (*P* < .0001) with laparoscopic partial nephrectomy versus open partial nephrectomy, while intraoperative complication rates were similar. Disadvantages of laparoscopic versus open partial nephrectomy were the significantly longer ischemia time (*P* < .0001) and the more frequent postoperative complications, especially urological disorders (*P* < .0001).

Importantly, the laparoscopic approach is associated with a reduction in postoperative pain and a shorter recovery period, posing surgeons and patients with a difficult decision between open and laparoscopic partial nephrectomies for a small incidentally detected renal tumor.

Renal laparoscopy will continue to develop, and urologists will gain greater experience with the technique over time. Thus, outcomes published by Gill et al. in 2007 were superior to those obtained by the same author in 2003 [41, 42]. It should be taken into account that the study by Gill et al. comparing laparoscopic nephrectomy with open partial nephrectomy [41, 43] was not a randomized clinical trial. In fact, most of the tumors selected for open partial nephrectomy were >4 cm, and all of them were centrally localized single tumors (size up to 7 cm) with a malignant histology. These cases are technically more challenging and carry a higher oncological risk, representing an important selection bias. There is a need for a randomized clinical trial to be undertaken to assess the risks and benefits of each approach. Nevertheless, there is an evident trend towards a minimally invasive approach to renal tumor treatment, and we can expect laparoscopic PN to develop in the near future to a point where it can replace open PN as a standard treatment for localized renal tumors.

At our center, we have treated 35 patients by conservative surgery of the renal parenchyma over the past 14 years (1993–2007), using open PN in 7 and enucleation in 28, with biopsies of the renal bed when involvement of the surgical margin was suspected. Indications were elective in 16 cases (45.5%), absolute in 11 (31.5%), and relative in 8 (23%). Mean size of tumors was 3.6 cm (range of 1–9 cm), with peripheral localization in 22 patients (63%), mesorenal in 12 (34%), and multifocal (6 tumors) in 1 patient (3%). Applying the technique described above in Section 5, we have had no intraoperative complications. Postoperative complications were renocutaneous fistula (resolved by internal derivation via ureteral catheter) and acute tubular necrosis (renal function recovered after hemodialysis) in the same single-kidney patient. After a median follow-up time of 69 months, we have observed one local recurrence (3%), which was from enucleation and was excised. Three patients died due to other causes and three were lost to the follow-up after moving from the area. All followed-up patients are disease-free and have creatinine levels similar to preoperative values.

Based on this experience, our group considers conservative renal surgery to be an alternative to radical surgery in tumors <4 cm or in larger tumors in single-kidney patients. Our selection of partial nephrectomy or enucleation is based on tumor localization and size. Thus, we prefer enucleation in tumors in mesorenal location because of its lower comorbidity versus PN. Our approach to peripheral tumors depends on their size. We use enucleation for small tumors of 1–3 cm, but we prefer partial nephrectomy for tumors ≥4 cm or when there is any suspicion of positive margins.

## 9. CONCLUSIONS

Open PN has been shown to be a safe and effective surgical technique in patients with a localized renal tumor, including patients with a normal contralateral kidney. We have gained experience with this technique by applying it to patients with an absolute indication, and we are now increasingly able to recommend it to patients with an elective indication, based on its good oncological outcomes and lower morbidity rates versus radical nephrectomy. Moreover, the preservation of nephrons achieved with open partial nephrectomy reduces the long-term risk of renal failure in these patients. These benefits outweigh any problems caused by the follow-up required for these patients due to fears of local recurrence, which will undoubtedly be more effectively detected at an earlier stage with new three-dimensional imaging techniques.

Nowadays, open PN is the gold standard technique to treat small renal masses, and all nonablative techniques must pass the test of time to be considered equally effective.

It is not ethical for patients to undergo radical surgery just because urologists involved do not have adequate experience with PN or have concerns about their capacity to manage its possible complications. Patients must be clearly informed about the possibility of laparoscopic PN in specialized centers. Patients should be involved in the final treatment decision and, when appropriate, referred to centers with experience in open or laparoscopic partial nephrectomies.

## Figures and Tables

**Figure 1:** Five-year survival: radical nephrectomy (RN) versus partial nephrectomy (PN).

**Figure 2:** Five-year disease-free survival by tumor size in patients undergoing partial nephrectomy.

**Figure 3:** Open partial nephrectomy for renal cell carcinoma of inferior pole satisfactory hemostasis with application of a fibrinogen hemostatic patch (Tachosil, Nycomed Pharma, Austria).

**Algorithm 1:** Indications for partial nephrectomy.

**Table 1:** Conservative renal surgery (partial nephrectomy); five-year outcomes in patients with elective indication.

Author, year	N	Disease-specific survival	Local recurrence	Mean tumor size
Morgan, 1990	20	100%	0%	3.1
Selli, 1991	20	90%	0%	3.5
Provet, 1991	19	100%	0%	2.6
Steinbach, 1992	72	94.4%	2.7%	ND
Moll, 1993	98	100%	1%	4
Lerner, 1996	54	92%	5.6%	4
D'Armiento, 1997	19	96%	0%	3.3
Van Poppel, 1998	51	98%	0%	3
Herr, 1999	70	97.5%	1.5%	3
Hafez, 1999	45	100%	0%	4
Barbalias, 1999	41	97.5%	7.3%	3.5
Belldegrun, 1999	63	100%	3.2%	4

**Table 2:** Complications after open partial nephrectomy.

Author, year (Hospital)	N	Acute renal failure (%)	Urinary fistula (%)
Ghavamian, 2002 (Mayo Clinic)	63	12.7	3.2
Duque, 1998 (Brigham)	64	15.1	9.1
Polascik, 1995 (Johns Hopkins)	67	1.5	9
Herr, 1994 (Memorial Sloan-KCC)	41	0	0
Campbell, 1994 (Cleveland Clinic)	259	12.7	17.3
